The article "Exploring Anti-Type 2 Diabetes Mellitus Mechanism of Gegen Qinlian Decoction by Network Pharmacology and Experimental Validation" was published in 2022. Journal: Dis Markers.

# Exploring Anti-Type 2 Diabetes Mellitus Mechanism of Gegen Qinlian Decoction by Network Pharmacology and Experimental Validation

**DOI:** 10.1155/2022/1927688

**Published:** 2022-10-15

**Authors:** Weiping Bao, Hongping Sun, Xiang Wu, Juan Xu, Huifeng Zhang, Lin Cao, Yaofu Fan

**Affiliations:** ^1^Department of Endocrinology, Affiliated Hospital of Integrated Traditional Chinese and Western Medicine, Nanjing University of Chinese Medicine, Nanjing, Jiangsu, China; ^2^Department of Geriatrics, Affiliated Hospital of Nanjing University of Chinese Medicine, Nanjing, Jiangsu, China

## Abstract

**Purpose:**

Gegen Qinlian Decoction (GGQL) has been employed to treat type 2 diabetes mellitus (T2DM) in the clinical practice of traditional Chinese medicine. However, the underlying mechanism of GGQL in the treatment of T2DM remains unknown. This study was aimed at exploring the pharmacological mechanisms of GGQL against T2DM via network pharmacology analysis combined with experimental validation.

**Methods:**

The effective components of GGQL were screened, and the target was predicted by using traditional Chinese medicine systems pharmacology database and analysis platform (TCMSP). The candidate targets of GGQL were predicted by network pharmacological analysis, and crucial targets were chosen by the protein-protein interaction (PPI) network. Gene Ontology (GO) and Kyoto Encyclopedia of Genes and Genomes (KEGG) functional enrichment analyses were performed to predict the core targets and pathways of GGQL against T2DM. Then, T2DM mice were induced by a high-fat diet combined with streptozotocin. The model and GGQL groups were given normal saline and GGQL aqueous solution (10 and 20 g/kg/d) intragastric administration, respectively, for 8 weeks. The mice in the GGQLT groups were administered with GGQLT at 10 and 20 g/kg/d, respectively. The pathological changes in liver tissues were observed by hematoxylin-eosin staining. The protein expression of TNF-*α* and NF-*κ*B was verified by western blotting.

**Results:**

A total of 204 common targets of GGQL for the treatment of T2DM were obtained from 140 active ingredients and 212 potential targets of T2DM. GO and KEGG enrichment analysis involved 119 signaling pathways, mainly in inflammatory TNF signaling pathways. Animal experiments showed that GGQL significantly reduced the serum levels of body mass, fasting blood glucose, fasting insulin, HOMA-IR, TNF-*α*, and IL-17. The liver pathological section showed that GGQL could improve the vacuolar degeneration and lipid deposition in the liver of T2DM mice. Mechanistically, GGQL downregulated the mRNA expression of TNF-*α* and NF-*κ*B.

**Conclusions:**

This study demonstrated that GGQL may exert antidiabetic effects against T2DM by suppressing TNF-*α* signaling pathway activation, thus providing a basis for its potential use in clinical practice and further study in treating T2DM.

The article "Exploring Anti-Type 2 Diabetes Mellitus Mechanism of Gegen Qinlian Decoction by Network Pharmacology and Experimental Validation" was published in 2022. Journal: Dis Markers.

## 1. Introduction

More than 90% of people with diabetes are type 2 diabetes mellitus (T2DM), whose pathological characteristics are mainly progressive beta-cell failure or insulin resistance (IR) [1, 2]. According to the International Diabetes Federation (IDF) Global Diabetes Map, the number of T2DM patients worldwide reached 463 million in 2021 [3]. It is estimated that by 2045, there are more than 700 million diabetes patients in the world, which would bring up a large economic burden on society [3]. The goals of diabetes management are to maintain their quality of life by keeping their blood sugar levels as close to normal as possible and within a target range and prevent or delay the development of various diabetic complications [4]. Over the past decades, a large number of glucose-lowering medications have been approved for clinical use in the control of T2DM, but most drugs have certain adverse reactions, such as hypoglycemia, gastrointestinal symptoms, oedema, osteoporosis, lactic acidosis, and urinary tract infection [5–7]. In addition, the management of complications of T2DM is still a major challenge in clinical practice and a substantial global healthcare burden [8]. Therefore, it is of necessity to explore the safe and effective anti-T2DM drugs for the clinical application.

Since ancient times, various medicinal plants were the first choice to treat diabetes as they are concerned with minimum side effects [9]. In recent years, large-scale clinical trials have confirmed that traditional Chinese medicine (TCM) has made progress in controlling blood glucose levels. An increasing number of studies have shown that Chinese formulae can be used in the prevention and treatment of diabetes through the “Bacteria-Mucosal Immunity-Inflammation-Diabetes” axis [10]. Gegen Qinlian Decoction (GGQL), which consists of *Radix puerariae*, *Radix scutellariae*, *Rhizoma coptidis*, and *Radix glycyrrhizae*, is a famous Chinese medicine prescription. GGQL was first recorded in a famous ancient medicine treatise Shanghan Lun, compiled by Zhong-Jing Zhang in the Han Dynasty of Chinese history (202 BC-220 AD). In previous researches, it has been found that GGQL exerts a range of pharmacological activities, including anti-inflammation, antidiabetic, antioxidant, and immunoregulative effects [11–14]. Our research team has confirmed that GGQL could decrease the fasting blood glucose (FBG) in mice with diabetes and improve the oral glucose tolerance and insulin tolerance in rats with T2DM [15]. These results indicate that GGQL has definite antidiabetic effects. However, the underlying pharmacological mechanisms of action of GGQL and its components in the treatment of T2DM remain unclear. More preclinical evidence is needed.

The article "Exploring Anti-Type 2 Diabetes Mellitus Mechanism of Gegen Qinlian Decoction by Network Pharmacology and Experimental Validation" was published in 2022. Journal: Dis Markers.

With the rapid progress of bioinformatics, systems biology, and polypharmacology, network pharmacology has been proven to be a novel strategy to elucidate the active compounds and potential mechanisms of TCM formulas. Therefore, this study was aimed at using network pharmacology to identify potential targets of GGQL as mediators of T2DM, thus providing useful clues for further experimental research. Mice fed a high-fat diet (HFD) combined with streptozotocin were used as a T2DM model to further explore the actions and mechanisms of GGQL against T2DM. This study provides a scientific basis for understanding the effectiveness of multicomponents, multitargets, and compound formulas as well as a new strategy for investigating therapeutic drugs for the treatment of T2DM.

## 2. Materials and Methods

### 2.1. Collection and Screening of Bioactive Compounds in GGQL

The active ingredients in GGQL were screened from the traditional Chinese medicine systems pharmacology database and analysis platform (TCMSP) (https://old.tcmsp-e.com/tcmsp.php) by using “Ge Gen”, “Huang Qin”, “Huang Lian”, and “Gan Cao” as keywords to identify targets related to GGQL. Oral bioavailability (OB) ≥ 30% and drug likeness (DL) ≥0.18 were employed to identify the potential active compounds in GGQL. With the help of the UniProt database (https://www.uniprot.org/), the effective compound composition information was converted into the corresponding target gene.

### 2.2. T2DM Disease Target Collection and Venn Diagram Construction

Using “T2DM” and “type 2 diabetes mellitus” as keywords, details on the human genes associated with T2DM were screened from GeneCards (http://www.genecards.org/), OMIM (https://omim.org/), PharmGkb (http://www.pharmgkb.org/), TTD (http://db.idrblab.net/ttd/), and DrugBank (http://www.drugbank.com/) databases. Repetitive targets were deleted, and all target genes were transformed into human genes by the UniProt database. The harvested GGQL-related targets and T2DM-related targets were subjected to a Venn diagram to determine the intersected targets.

### 2.3. Construction of GGQL Component-T2DM-Target Interaction Network and Protein-Protein Interaction (PPI) Network

The GGQL-compound-target-T2DM network was constructed by Cytoscape 3.8.2. As previous researches show, intersection targets were imported into the STRING 11.0 database (https://string-db.org/). Species were positioned as “Human,” and the confidence threshold was set as >0.90. The selected proteins were introduced into Cytoscape 3.8.2 software to construct PPI networks, and the node connectivity was analyzed to screen out the core targets.

The article "Exploring Anti-Type 2 Diabetes Mellitus Mechanism of Gegen Qinlian Decoction by Network Pharmacology and Experimental Validation" was published in 2022. Journal: Dis Markers.

### 2.4. Gene Ontology (GO) Functional Annotation and Kyoto Encyclopedia of Genes and Genomes (KEGG) Pathway Analysis

R software, a free software environment for statistical computing and graphics, was used to perform GO and KEGG functional enrichment analyses for the key targets. The threshold value was *P* < 0.05. GO analysis analyzed the functional level of potential target genes from three aspects: biological process (BP), cell composition (CC), and molecular function (MF). KEGG analysis showed that GGQL interfered with the biological pathway of T2DM. The top 10 items of GO analysis and the top 20 items of KEGG analysis identified from R software were mapped as bubble plots.

### 2.5. Animal

40 C57BL/6J mice, male, SPF grade, 12 weeks old, were purchased from Shanghai Shrek Experimental Animal Co., Ltd., license number: SCXK (Shanghai) 2017-0005, feeding condition, relative humidity 50%, Mel 70%. The feeding and experimental process of the animals involved in the experiment followed the relevant guidelines for the management and protection of experimental animals in the Hospital of Integrated Traditional Chinese and Western Medicine affiliated to Nanjing University of Traditional Chinese Medicine (reference number: AEWC-20190814-81).

### 2.6. Drugs, Reagents, and Instruments

All pieces of traditional Chinese medicine in GGQL were purchased from the Hospital of Integrated Traditional Chinese and Western Medicine affiliated to Nanjing University of Traditional Chinese Medicine. The quality ratio of Gegen (batch number: 20170301), Huangqin (batch number: 1610009), Huanglian (batch number: 1703015), and Gancao (batch number: 170109) was prepared according to the ratio of 8 : 3 : 3 : 2. The preparation of GGQL was made according to the method described in the literature [16]. Pioglitazone hydrochloride tablets (batch number H20110048, Jiangsu Deyuan Pharmaceutical Co., Ltd.). The tumor necrosis factor-*α* (TNF-*α*) and interleukin-17 (IL-17) ELISA kits were purchased from Jiangsu Biyuntian Biotechnology Co., Ltd.; the TNF-*α*, nuclear factor kappa-B (NF-*κ*B), and *β* actin antibodies were purchased from the American Abcam company; and the second anti-rabbit was purchased from the American CST company. The biospectrum-gel imaging system was from Bio-Rad company, USA; tissue slicer from Leica company, Germany; and optical microscope from Olympus company, Japan.

### 2.7. Modeling and Drug Delivery

After 1 week of adaptive feeding, 40 C57BL/6J mice were randomly divided into a normal fat diet group (NFD group, *n* = 8) and HFD group (*n* = 32). The HFD group was fed with high-fat diet (purchased from Nantong Tolofei Feed Technology Co., Ltd., batch number 2017416, with a formula of 60% high-fat model feed). After 4 weeks of feeding, 1% streptozotocin solution 45 mg kg-^1^ was injected intraperitoneally (lasting 3 days). 72 hours after injection, random blood glucose ≥ 16.7 mmol/L was detected in the tail vein, and T2DM modeling was successful. HFD group mice were equally divided into 4 groups: HFD group (received saline 10 ml/kg/d), pioglitazone group (PIO group, received pioglitazone 30 mg/kg/d), low-dose GGQL group (GGQLL group, received GGQL 10 mg/kg/d), and high-dose GGQL group (GGQLH group, received GGQL 20 mg/kg/d). The NFD group was also administrated with saline (10 ml/kg/day). All these doses were given via oral gavage daily for 8 weeks. The weight of mice was weighed every week to adjust the dose of intragastric administration.

The article "Exploring Anti-Type 2 Diabetes Mellitus Mechanism of Gegen Qinlian Decoction by Network Pharmacology and Experimental Validation" was published in 2022. Journal: Dis Markers.

### 2.8. Biochemical Analysis and Histopathological Examination

At the end of the experiment, abdominal aortic blood samples were taken after the last dose. The serum sample was used to measure the levels of FBG. Kits were purchased from Nanjing Jiancheng Bioengineering Institute (Nanjing, China). The plasma insulin (FINS), TNF-*α*, and IL-17 were measured by ELISA Assay Kit (ALPCO, USA). Homeostasis model assessment of insulin resistance index (HOMA-IR) was calculated using the previously described formula: HOMA‐IR = FINS × FBG/22.5. 10% formalin-fixed liver tissues were embedded in paraffin, cut into 4 *μ*m thick sections, and then stained with hematoxylin and eosin (H&E) for histopathological examination. Sections were examined, and digital pictures were captured using an Olympus digital camera (BX20, Beijing, China) using NIS Element SF 4.00.06 software (Beijing, China) and photographed at 200× magnification for analysis.

### 2.9. Western Blotting

Western blotting analysis of proteins was carried out as previously reported [15]. The liver tissue of 100 mg was homogenized, and the total protein was extracted according to the instructions of the whole protein extraction kit. The concentration of total protein was determined by BCA kit, and the same amount of protein was electrophoretic by 10%SDS-PAGE. After being transferred to polyvinylidene fluoride (PVDF) membrane, 5% skim milk was used to seal the protein at room temperature for 2 hours. Protein gel electrophoresis was carried out according to the western blot method, and a gel imaging analysis system was used to detect protein bands.

### 2.10. Statistical Analysis

All data were expressed as mean ± SEM. Results were tested for normal distribution, then were analyzed using ANOVA followed by Bonferroni post hoc test using GraphPad Prism 5.01 (GraphPad Software Inc., San Diego, CA, USA). *P* values < 0.05 were considered as statistically significant.

The article "Exploring Anti-Type 2 Diabetes Mellitus Mechanism of Gegen Qinlian Decoction by Network Pharmacology and Experimental Validation" was published in 2022. Journal: Dis Markers.

## 3. Results

### 3.1. GGQL Active Compound Network Analysis

GGQL obtained a total of 146 chemical components after searching the TCMSP database, with 4 compounds from Gegen, 36 compounds from Huangqin, 14 compounds from Huanglian, and 92 compounds from Gancao. There are 140 components after deleting the duplicate value, and the top 20 items of active components are shown in Table 1. Correcting based on the UniProt database, we obtained 212 targets in total.

### 3.2. Potential GGQL Targets Treat T2DM and Network Analysis

To elucidate the mechanism and pharmacodynamics of GGQL, 10821 target genes of T2DM were obtained from GeneCards, OMIM, PharmGkb, TTD, and DrugBank databases. Further analysis with Venn diagrams identified 204 targets associated with both T2DM and GGQL that are displayed in Figure 1(a). Then, to elucidate the relationship between active ingredients and potential targets as well as T2DM, an ingredient-target-disease network was constructed by Cytoscape 3.8.2 software, consisting of 349 nodes and 1989 edges (Figure 1(b)). The top 10 key active ingredients of GGQL in the treatment of T2DM are enumerated in Table 2.

### 3.3. PPI Network Construction and Key Targets

To elucidate the potential mechanism by which GGQL protects against T2DM, PPI relationships of the 204 target genes were obtained using the STRING tool, and the results are displayed in Figure 2(a). Then, we used the Cytoscape software to calculate the topological parameters, and 18 core targets were obtained. The top 10 key targets in the core position were JUN, AKT1, STAT3, MAPK3, FOS, MAPK1, MYC, MAPK14, ERS1, and TP53, as shown in Figure 2(b).

### 3.4. Pathway and GO Term Enrichment Analysis

The drug-disease common targets were processed by R language for GO function and KEGG pathway enrichment analysis. The GO enrichment bubble chart was formed by selecting the top 10 significant biological process (BP), cellular components (CC), and molecular function (MF), as shown in Figure 3.

To explore the signal pathway mechanism of GGQL in the treatment of T2DM, we performed KEGG enrichment analysis. As shown in Figure 4, it shows the first 20 signal pathways, which involve the TNF signaling pathway, IL-17 signaling pathway, and so on. The key KEGG pathway and the location of T2DM and overlapping genes of enriched pathways are listed in Figure 5.

### 3.5. GGQL Ameliorated IR in HFD Mice

Figure 6(a) shows that within HFD-fed mice, treatment with GGQLL or GGQLH could alter body weight compared with HFD mice, but these were not statistically significant. The HFD-fed group mice led to a marked elevation in the levels of fasting glucose, fasting insulin, and HOMA-IR in the serum region compared with those of the control group, as shown in Figures 6(b)–6(d).

The article "Exploring Anti-Type 2 Diabetes Mellitus Mechanism of Gegen Qinlian Decoction by Network Pharmacology and Experimental Validation" was published in 2022. Journal: Dis Markers.

### 3.6. Effects of GGQL on Hepatic Tissue

The HE staining of the liver tissue of mice in each group is shown in Figure 7. The results showed that, compared with the NFD group, lipid deposition, vacuolar degeneration, and watery degeneration were observed in the liver of the HFD group.

### 3.7. Effects of GGQL on the TNF Signaling Pathway in T2DM Mice

The network pharmacology results demonstrated that the potential targets of GGQL against T2DM were significantly enriched in the TNF pathways. Compared with the NFD group, the expression of TNF-*α* and NF-*κ*B in the HFD group increased, while the expression of TNF-*α* and NF-*κ*B in the GGQLL, GGQLH, and PIO groups decreased significantly compared with that in the HFD group (all *P* < 0 01) (Figure 8).

## 4. Discussion

The incidence of T2DM has been rising in recent years due to the aging of the population and changes in lifestyle [17, 18]. Currently, oral antidiabetic drugs are mainly focused on a single compound and reported to have adverse effects [19]. TCM has a rich history and has shown good results in the treatment of T2DM. Hence, TCM may be a prospective option for T2DM intervention. Due to TCM's effectiveness depending on multitarget and multicomponent, it is difficult to explore its mechanism of action. This study draws lessons from the research ideas of network pharmacology, through the analysis of various networks to identify multicomponents and multitargets involved in the treatment of T2DM by GGQL.

According to the network pharmacology analysis, we obtained 140 active compounds from GGQL that acted on 212 targets of T2DM. The active compounds were mainly flavonoids. According to the degree value, the top three active ingredients were quercetin, kaempferol, and wogonin. Quercetin is a natural polyhydroxyflavone, which can reduce the level of oxidative stress, inhibit apoptosis of INS-1 cell, and promote insulin secretion [20]. A large cross-sectional study in China showed that quercetin intake was negatively correlated with the prevalence of T2DM [21]. Kaempferol can increase the activities of AKT and hexokinase, decrease the activity of glucose-6 phosphatase in the liver, and play a hypoglycemic effect by inhibiting gluconeogenesis in the liver [22]. Wogonin can promote glucose uptake and glycolysis through the insulin receptor-1/PI3K/alkaline phosphatase pathway, inhibit gluconeogenesis in hepatocytes, and improve insulin resistance [23]. Therefore, all of these findings showed that multiple components of GGQL had a positive effect on T2DM.

18 key genes were screened by constructing PPI network and performing network topology structure with Cytoscape software, including JUN, AKT1, and STAT3. JUN is an important signal molecule connecting inflammation and insulin resistance. Studies have confirmed that high glucose-induced apoptosis can be inhibited by inhibiting the JUN signal pathway [24, 25]. Increasing the expression of AKT1 in islet cells can reduce islet cell apoptosis and increase secretory function [26, 27]. STAT3, a signal transducer and activator of transcription 3, is highly expressed in T2DM patients. Animal studies have found that inhibiting the expression of STAT3 in obese rats can prevent the development of lipid-induced insulin resistance and reduce the incidence of diabetes [28, 29].

The article "Exploring Anti-Type 2 Diabetes Mellitus Mechanism of Gegen Qinlian Decoction by Network Pharmacology and Experimental Validation" was published in 2022. Journal: Dis Markers.

In addition, the GO enrichment analysis showed that the pharmacological effects of GGQL on T2DM were related to TNF signaling. The target points in the KEGG enrichment analysis were also enriched in the TNF-*α* signaling pathway. In recent years, with the in-depth study of the pathogenesis of T2DM, many scholars believe that T2DM may be an immune inflammatory disease, in which TNF-*α* is involved in the regulation of inflammatory response and glucose and lipid metabolism [30, 31]. Skuratovskaia et al. found that TNF-*α* can inhibit the phosphorylation of insulin receptor substrate-1, which leads to insulin resistance in liver and adipocytes, and increases the progression of T2DM [32]. In addition, a previous study has shown that TNF-*α* can not only induce the occurrence of diabetes but also cause damage to vascular endothelial function, initiate the process of atherosclerosis, and increase the risk of various complications of diabetes [33]. All the above studies have shown that the TNF-*α* signaling pathway plays an important role in T2DM. Animal experiments showed that GGQL can effectively reduce the levels of insulin, HOMA-IR, TNF-*α*, and IL-17 and improve the state of hyperglycemia. We also found that the protein expression levels of TNF-*α* and NF-*κ*B in the liver tissues of HFD mice were significantly increased, While GGQL could restore them. Many other scholars' studies are consistent with our findings. Xu et al. found that GGQL suppressed activation of NF-*κ*B and TNF-*α* to inhibit T2DM development [14]. Li et al. revealed that GGQL could reduce the TLR4 expression and NF-*κ*B activation along with several inflammatory cytokines such as TNF*α* and IL-6 [34].

However, there are still several limitations in our study to be solved in the future work. One was the study only performed in vivo experiments, which lacked corresponding cellular experiments to validate the function and mechanism of GGQL on T2DM. In the future, we will conduct cellular experiments to better prove the results. Second, we only explored one pathway that we think is more likely to work. As we did not verify other possible pathways, we cannot verify whether GGQL can participate in other pathways to make a synergistic antidiabetic effect. Third, although the TNF-*α* signaling pathway was verified to be involved in mechanism of action, the potential upstream or downstream relationships between TNF-*α* still need to be further explored.

The article "Exploring Anti-Type 2 Diabetes Mellitus Mechanism of Gegen Qinlian Decoction by Network Pharmacology and Experimental Validation" was published in 2022. Journal: Dis Markers.

## 5. Conclusions

In the present study, we combined network pharmacology prediction and in vivo experiments to research the active ingredients, potential targets, and potential mechanism of GGQL against T2DM. The results suggest that GGQL ameliorates blood sugar by improving IR and inhibiting inflammation. These effects appear to be related to GGQL affecting the TNF-*α* signaling pathways. This work supplies a foundation for the treatment of endocrine disorder-related complex diseases with TCM and lays a certain theoretical foundation for further exploration to expand the application of GGQL. Detailed pharmacological mechanisms by which GGQL ameliorates T2DM will be investigated in our future study.

## Figures and Tables

**Figure 1:** Potential GGQL targets treat T2DM and network analysis. (a) Venn diagram summarizing the intersection targets of the GGQL and T2DM. (b) Network of targets shared between GGQL and T2DM. The ring represented the composition, and the rectangle represented target genes.

**Figure 2:** PPI network construction and key targets. (a) PPI network of potential targets of GGQL for the treatment of T2DM. (b) Obtaining 18 core proteins of GGQL for T2DM.

**Figure 3:** Top 10 GO terms of hub genes.

**Figure 4:** Top 30 KEGG pathways of hub genes.

**Figure 5:** The key KEGG pathway: TNF signaling pathway. The red nodes represent overlapping targets between GGQL and T2DM.

**Figure 6:** (a) Body weight was measured every week during the treatment period. The expression of serum (b) glucose and (c) insulin concentration. (d) HOMA-IR was calculated at the end of the experiment. ^∗^*P* < 0.05; ^##^*P* < 0.01. Data are expressed as the means ± SEM of at least three independent experiments.

**Figure 7:** Effects of GGQL on hepatic pathological changes. Histological observation of the hematoxylin and eosin (H&E) sections (original magnification ×400). Macrovesicular steatosis was observed in the livers of mice.

The article "Exploring Anti-Type 2 Diabetes Mellitus Mechanism of Gegen Qinlian Decoction by Network Pharmacology and Experimental Validation" was published in 2022. Journal: Dis Markers.

**Figure 8:** Western blot and densitometric analysis of the expression of TNF-*α*, NF-*κ*B, and *β*-action in mice. ^∗∗^*P* < 0.01 compared to the NFD group, which was considered statistically significant.

**Table 1:** Active components of GGQL (top 20 of OB).

Mol ID	Active components	OB (%)	DL
MOL002907	Corchoroside A_qt	104.95	0.78
MOL002934	Neobaicalein	104.34	0.44
MOL002311	Glycyrol	90.78	0.67
MOL008647	Moupinamide	86.71	0.26
MOL004990	7,2′,4′-Trihydroxy-5-methoxy-3-arylcoumarin	83.71	0.27
MOL004904	Licopyranocoumarin	80.36	0.65
MOL004891	Shinpterocarpin	80.3	0.73
MOL005017	Phaseol	78.77	0.58
MOL004841	Licochalcone B	76.76	0.19
MOL002932	Panicolin	76.26	0.29
MOL004810	Glyasperin F	75.84	0.54
MOL001484	Inermine	75.18	0.54
MOL000500	Vestitol	74.66	0.21
MOL012246	5,7,4′-Trihydroxy-8-methoxyflavanone	74.24	0.26
MOL005007	Glyasperins M	72.67	0.59
MOL004941	(2R)-7-Hydroxy-2-(4-hydroxyphenyl) chroman-4-one	71.12	0.18
MOL004959	1-Methoxyphaseollidin	69.98	0.64
MOL000392	Formononetin	69.67	0.21
MOL002927	Skullcapflavone II	69.51	0.44
MOL002911	2,6,2′,4′-Tetrahydroxy-6′-methoxychaleone	69.04	0.22

**Table 2:** The top 10 key active ingredients of GGQL in the treatment of T2DM.

Molecular ID	Ingredient	Degree	Source	OB (%)	DL
MOL000098	Quercetin	135	Gancao	46.43	0.28
			Huanglian		
MOL000422	Kaempferol	54	Gancao	41.88	0.24
MOL000173	Wogonin	40	Huangqin	30.68	0.23
MOL003896	7-Methoxy-2-methyl isoflavone	35	Gancao	42.56	0.20
MOL004328	Naringenin	34	Gancao	59.29	0.21
MOL002714	Baicalein	31	Huangqin	33.52	0.21
MOL000392	Formononetin	30	Gancao	69.67	0.21
			Gegen		
MOL000497	Licochalcone A	30	Gancao	40.79	0.29
MOL000354	Isorhamnetin	29	Gancao	49.60	0.31
MOL002565	Medicarpin	26	Gancao	49.22	0.34

## Data Availability

The data are available upon direct request to the corresponding authors.
